The article "Occurrence of Total Aflatoxins, Aflatoxin B1, and Ochratoxin A in Chicken and Eggs in Some Cameroon Urban Areas and Population Dietary Exposure" was published in 2022. Journal: J Environ Public Health.

# Occurrence of Total Aflatoxins, Aflatoxin B_1_, and Ochratoxin A in Chicken and Eggs in Some Cameroon Urban Areas and Population Dietary Exposure

**DOI:** 10.1155/2022/5541049

**Published:** 2022-06-11

**Authors:** Fabrice De Paul Tatfo Keutchatang, Alex K. Tchuenchieu, Evelyne Nguegwouo, Hippolyte Tene Mouafo, Isabelle Sandrine Bouelet Ntsama, Germain Kansci, Gabriel Nama Medoua

**Affiliations:** ^1^Centre for Food and Nutrition Research, Institute of Medical Research and Medicinal Plants Studies, P.O. Box 6163, Yaoundé, Cameroon; ^2^Department of Biochemistry, Laboratory of Food Science and Metabolism, Faculty of Sciences, University of Yaoundé I, P.O. Box 812, Yaoundé, Cameroon; ^3^Food Evolution Research Laboratory, School of Tourism and Hospitality, College of Business and Economics, University of Johannesburg, Johannesburg 2000, South Africa; ^4^Advanced Teacher's Training College for Technical Education, University of Douala, P.O. Box 1872, Douala, Cameroon

## Abstract

Consumption of chicken and eggs contaminated by mycotoxins could lead to a public health concern. This study was conducted to evaluate the dietary exposure of populations to aflatoxins (AFs) and ochratoxin A (OTA) through these poultry products in the three most urbanized regions of Cameroon (Centre, Littoral, and West). A survey was firstly carried out to know about the consumption frequency by the different population age groups as well as their awareness about mycotoxins. Chicken feed, broiler, and eggs were collected from modern poultry farms. AFs and OTA were analysed using the enzyme-linked immunosorbent assay (ELISA), and dietary exposure was evaluated using a deterministic approach. From the 900 households questioned, a daily consumption frequency of chicken and eggs was the most reported (41% and 69%, respectively), with populations having a very weak knowledge of mycotoxins and their associated health risk (18%). Mean concentrations of AFs, AFB_1_, and OTA in poultry tissues were below the established regulated limits (20 *μ*g/kg for AFs, 10 *μ*g/kg for AFB_1_, and 5 *μ*g/kg for OTA) in feeds. These toxins were detected at average concentrations of 1800 and 966.7 *ƞ*g/kg for AFs in chicken muscle and egg, respectively, and 1400 and 1933.3 *ƞ*g/kg for OTA in muscle and egg, respectively. Based on the survey, their estimated daily intakes through these poultry products tended to be lower than the limits 1 and 100 *ƞ*g/kg bw/day for AFB_1_ and OTA, respectively). The margins of exposure (MOE) of the different population age groups to AFB_1_ and OTA obtained suggest that the public health concern associated with the presence of mycotoxins in poultry products shall not be underestimated.

## 1. Introduction

Poultries such as chicken are important sources of protein and other nutrients for human nutrition [1]. Chicken is easy to rear [2], available at low prices, and consumed by billions of people including those who live in low-income countries [3]such as Cameroon. In 2018, 69 billions of chickens were killed and processed for meat around the world [4]. The poultry sector is a growing industry that accounts for about 33% of the global meat consumption and is expected to increase at 2-3% per year in the world [5]. In Cameroon, it has been estimated to share 42% of the market with a per capita consumption of 5.6 kg of chicken and 52 eggs annually [2]. Poultry feed generally consists of agricultural products such as maize, groundnuts, and wheat that may be contaminated by mycotoxins. Several studies reported the poisoning of humans and animals caused by feed and food contaminated by mycotoxins [6–9]. These mycotoxins have been described as carcinogenic, nephrotoxic, hepatotoxic, teratogenic, and immunotoxic to humans and several other species of animals [10]. They are a group of secondary metabolites produced by fungi belonging to three genera (*Aspergillus, Penicillium*, and *Fusarium*) which can produce more than 500 toxins. Amongst these mycotoxins, some like aflatoxins and ochratoxin A exhibit pathogenic characteristics [8, 9]. They are nowadays considered as a worldwide concern by the WHO and FAO. In suitable conditions, fungal growth in animal feed is inevitable (especially during storage). The use of contaminated feed in the poultry sector is a source of cross-contamination for humans. Human exposure to these mycotoxins is generally more important through plant food than animal food, but regular consumption of animal products even if containing low mycotoxins levels may lead to health problems. In Cameroon, previous studies reported the contamination of chicken feed by mycotoxins [11, 12] and their occurrence in gizzard, chicken muscle, and eggs [13, 14]. However, to the best of our knowledge, no study has been carried out to assess the dietary exposure that could be associated with the presence of these toxins in chicken and eggs which are frequently consumed. The present study was designed to assess the occurrence of total aflatoxins, aflatoxin B_1_, and ochratoxin A in chicken and eggs and the associated health risk for the different population age groups.

## 2. Materials and Methods

### 2.1. Study Design and Survey Data Collection

A survey on chicken and eggs consumption and population awareness about mycotoxins was firstly carried out. This was a cross-sectional, multistage cluster study conducted in three regions of Cameroon (Centre, Littoral, and West).  Figure 1 presents the distribution of the study clusters. Thirty clusters were selected in each region using a random start point and systematic selection of adjacent households, each cluster representing 10 households. A total of 900 voluntary households took part in this survey, with as inclusive criteria a minimum of 2 years of settlement of the concerned family in the area. The household respondents should also have at least 18 years old. The questionnaire was drafted (and validated in 20 households) to collect information regarding people living in the house (age, weight), their chicken and egg consumption frequency as well as quantity, and their knowledge of fungi and mycotoxins. Chicken and egg consumption frequency and quantities were assessed by asking participants how many times in the week, month, or year they had consumed chicken or eggs and the number of eggs or parts of the chicken generally eaten by each member of the household. An estimation of the corresponding weight could therefore be made by removing the bias associated with the presence of the bones in the chicken part (averagely 71.1% of a part) and eggshells (averagely 12.8% of an egg) that are not eaten. Wearing minimal clothes, the elderly, adults, teenagers, and children of each household were weighed to the nearest 10 g with an electronic scale (Seca, Hamburg, Germany).

### 2.2. Sample Collection

Fifteen samples of chicken feed, 48 live market-ready broilers, and 180 fresh layer eggs were randomly collected as described by Akinmusire et al. [15] for feed samples and Thrusfield [16] for other samples. Indeed, sampling was conducted in 6 different poultry farms (2 per region) for broilers, 6 other layer farms (2 per region) for chicken eggs, and 12 poultry farms (the previous 6 for broilers and 6 for layers) and in 3 commercial structures for chicken feeds (local and imported feed). The samples collected were brought to the laboratory for treatments and analyses.

### 2.3. Sample Treatments

Feed samples were ground with a blender (Black & Decker®; England), weighed in several aliquots of 5 g using a scale (Mettler Tolero, USA), and stored in sterile plastic bags at −20 C until analysis (maximum 1 week). Chicken samples were slaughtered, and their carcasses were scalded using hot water at 100 ± 2 C. The skeletal muscle, as well as the skin and liver of each broiler, were removed with a knife. The most consumed parts such as the muscle and the liver were taken from each broiler to make a bulk sample of each part for a broiler farm. Each bulk sample was ground separately and thoroughly mixed to give representative samples. Ground bulk samples were weighed in several aliquots of 5 g and stored at −80 C until analysis. Eggs samples were washed with distilled water, broken, homogenized, weighed in several aliquots of 5 g, and also stored at −80 C until analysis.

### 2.4. Mycotoxin Determination

Total aflatoxins (AFs), aflatoxin B_1_ (AFB_1_), and ochratoxin A (OTA) concentrations in the samples were determined using quantitative ELISA (enzyme-linked immune sorbent assay) kits (CAT. No. 1030, 1034 and 1036, BIOO Scientific Corp., MaxSignal®, Burleson Road Austin, TX 78744 USA). Samples (5 g of chicken feed, 2 g of ground bulk chicken tissue, or 2 g of egg) were mixed with 25 mL of 70% methanol (HPLC grade Merck) in 50 mL falcon tubes for 10 min on a vortex, followed by centrifugation at 4,000 ×g for 10 min using the Rotofix 32 A, centrifuge (Germany). Then, 100 *μ*L of the supernatant was collected and diluted with 700 *μ*L of a mixture of methanol (HPLC grade, Merck). The mixture was used for total AFs, AFB_1_, and OTA analyses following the kit manufacturer's instructions. Their concentrations were inversely proportional to the colour intensity established using an automated microplate reader (EL × 800, BIOTEK, Instruments Inc., Winooski, VT, United States) at 450 nm and were estimated based on a calibration curve plotted before. The analytical test was evaluated using the internal quality control (IQC) approach and validated before usage. Five different IQCs were chosen to monitor the analytical sequence: calibration, blanks, midrange standard, spiked standard solution, certified references material, and duplicates. When acceptance criteria were not met for a sample, results were discarded, and the sample was reanalysed. The limit of detection (LOD) of the analysed samples varied between 0.06–0.3 *μ*g/kg for AFs and 0.3–0.6 *μ*g/kg for OTA, while the limit of quantification (LOQ) was in the range 0.2–1 *μ*g/kg for AFs and 1–2 *μ*g/kg for OTA. Samples with values below the limit of quantification (LOQ) were recorded as containing not detectable.

### 2.5. Dietary Exposure Assessment

A deterministic approach was used to calculate dietary exposure to AFT, AFB_1_, and OTA [17]. Amongst aflatoxins, AFB_1_ is the most dangerous and is known with OTA to be heat stable at 160°C and 180°C, respectively [18]. Their intakes were determined by considering the mean concentrations of mycotoxins and the min, mean, max, and 95th percentile of the collected chicken and egg consumption. The following equation was used:

(1) $$\begin{array}{c} \text{daily dietary exposure to AFT or }{\text{AFB}}_{1}\text{or OTA}=\\ \frac{\text{amount of chicken or eggs daily consumed for each individual group}\left(\text{g}/\text{day}\right)\times {\text{AFB}}_{1\;}\text{ or OTA concentration }\left(\mu \text{g}/\text{kg}\right)}{\text{body weight}\left(\text{kg}\right)}. \end{array}$$

The risk was majored as we assumed that the mycotoxins are not destroyed during the cooking process. To estimate the daily dietary exposure, the average body weights of children, teenagers, adults, and elderly people were considered as well as the quantity of chicken and eggs daily consumed. The margins of exposures (MOEs) to the studied mycotoxins were calculated as a ratio of the benchmark dose low limit 10% lower bound (BMDL_10_) of the toxin and the estimated toxin intake divided by 1000 [19, 20]. The BMDL_10_ represents the lowest dose with a 95% certainty of not leading to a 10% increase in cancer incidence in rodents and was fixed at 400 *ƞ*g/kg bw/day and 17.86 *ƞ*g/kg bw/day for AFB_1_ and OTA, respectively [20–23]. Dietary intake from chicken was calculated using the average concentration of AFT, AFB_1_, and OTA obtained in the muscle and the liver.

### 2.6. Data Analysis

Data obtained from survey and mycotoxin analysis were compiled in a database system using Microsoft Excel software. Descriptive statistics were performed to summarize data as the mean ± standard deviation (SD) for continuous variables and percentages for categorical variables. The Pearson correlation coefficient was used to evaluate the relationship between the tested variables using SPSS 20.0. Variables with *p* < 0.05 were considered significant at 95% confident interval (CI).

## 3. Results and Discussion

### 3.1. Chicken and Egg Consumption and Consumers' Knowledge about Mycotoxins

Amongst the 900 household respondents, 61.3% respondents were women and 38.7% were men (Table 1). Their level of studies mainly ranged from primary (13.7%) to university (47.3%), 34.3% having a secondary school level. The Centre region registered the highest percentage of respondents with just a primary level of study (21%), the Littoral region, the highest percentage of respondents who had secondary level of study (54%), and the West region, the highest percentage of those with a university level of study (59%). Up to 95.7% of the total population studied had a general knowledge of moulds, but 77.0% of the population did not know that mould contamination may imply the presence of mycotoxins. Respondents from the Littoral region were more informed about fungal contamination (98%) but were less aware of the associated health risks (2%). On the contrary, the respondents in the West region were less aware of fungal contamination (93%) but more aware about the associated health risks (29%). Only 18.0% of all the 900 respondents affirmed that health risk could be linked to fungal contamination. A similar percentage (12%) was reported by Nguegwouo et al. in 2018 [24] when questioning 100 persons living in the Centre region (Yaoundé) about their knowledge of moulds and mycotoxins. A significant correlation between the education level and this knowledge was noticed (*p* < 0.05). This survey globally revealed a daily consumption of chicken and eggs, the highest percentage being recorded in the Centre region (45%) for daily chicken consumption and in the West region (72%) for daily egg consumption. Data from this survey led to an estimation of the mean body weight of chicken and egg consumers of 25.2 ± 5.2 kg for children (4–12 years old), 56.3 ± 6.0 kg for teenagers (13–20 years old), 71.4 ± 10.2 kg for adults (21–59 years old), and 76.9 ± 7.7 kg for elderly people (≥60 years old) (Table 2). The estimated daily consumption average varies from 12.5 g (children) to 85.9 g (elderly people) for chicken, while for eggs it ranges from 15.5 g (children) to 48 g (teenagers). Considering the average consumption levels of each individual group, they are higher than the per capita consumption levels of poultry and eggs reported in the country in 2006 by Teleu and Ngatchou [25] (10.9 g/day (4 kg/year) and 2.5 g/day (0.9 kg/year), respectively, and the 9.81 g cooked/day for poultry and 7.15 g cooked/day for eggs obtained during the second Cameroonian Household Budget Survey (HBS/ECAM II) in 2001 [26].

### 3.2. Mycotoxin Contents of the Samples

AFs, AFB_1,_ and OTA were detected in all chicken feed, chicken tissues, and eggs (Table 3). Concerning chicken feed samples, they globally respected the standard recommended. Indeed, AFs were found in a range that varies between 3500 and 19700 *ƞ*g/kg, which is below the maximum tolerable limit of 20 *μ*g/kg (20000 *ƞ*g/kg) [27]. This is lower than values reported in previous studies in Guyana (27380 ± 82120 *ƞ*g/kg; [28]), Nigeria (127400 *ƞ*g/kg; [15]), and Cameroon (30000 and 22000 *ƞ*g/kg; [11]). Aflatoxin B_1_ was also found in all chicken feed samples in an average concentration of 1500–19300 *ƞ*g/kg. However, just 2 samples over the 13 feed samples tested (2/13) showed concentrations above the regulatory limit which are 10 *μ*g/kg (10000 *ƞ*g/kg) [29]. This is probably the consequence of conditions in which feed samples are produced or stored which promote this toxin production by moulds such as *Aspergillus* of which presence has already been reported [30]. The OTA concentrations detected in all chicken feed (800–2400 *ƞ*g/kg) were also below the maximum tolerable limit of 5 *μ*g/Kg (5000 *ƞ*g/kg) [29]). Previous studies in Nigeria and Cameroon had already reported the contamination of chicken feed or poultry by OTA at variable concentrations (1200 and 2100 *ƞ*g/kg [11]; 5400 *ƞ*g/kg [15]). Mycotoxins can be carried over from feed to the animal body and be bioaccumulated [31]. The studied mycotoxins (AFs, AFB_1_, and OTA) were also found in bulk chicken muscle, liver and egg samples. For aflatoxins, the level of AFB_1_ in chicken samples (700–1200 *ƞ*g/kg) and eggs (800–1100 *ƞ*g/kg) was close to the total AFs levels observed (1400–2500 *ƞ*g/kg and 700–1900 *ƞ*g/kg, respectively). Hopefully, the concentrations detected respect the maximum tolerable level of 2 *μ*g/kg (2000 *ƞ*g/kg) for AFB_1_ in human food products set by the European Commission and many other countries [32]. Considering the potentially toxic effects of AFs and OTA, their concentration in chicken products for human consumption has to follow the ALARA principle to preserve human health [33]. Ochratoxin A was noticed at the average concentrations of 1400 ± 173.2 *ƞ*g/kg for bulk muscle; 2266.7 ± 1000 *ƞ*g/kg for bulk liver, and 1933.3 ± 208.2 *ƞ*g/kg for bulk layer eggs. This higher presence of OTA in the liver than in the muscle was not observed with AFs but may be explained by the fact that liver is the organ where mycotoxins are metabolized [34]. The presence of these mycotoxins in chicken tissues and eggs had already been reported in previous studies [13, 35]. These results corroborate the report of Pouokam et al. [35] in 2017 according to which foods of animal origin also faced significant contamination from various contaminants, including mycotoxins.

### 3.3. Exposure Level of the Population to Aflatoxin B_1_ and OTA

Based on the AFT, AFB_1_, and OTA contamination levels observed in chicken tissues and eggs as well as the consumption of these foods collected, the daily intake (min, max, mean, and percentiles 75 and 95) of the toxins analysed were determined (Table 4). The estimated average daily dietary exposures (EDE) to AFT and AFB_1_ through chicken consumption were found to be, respectively, 0.9 and 0.6 *ƞ*g/kg bw/day for children, 1.3 and 0.8 *ƞ*g/kg bw/day for teenagers, 0.7 and 0.4 *ƞ*g/kg bw/day for adults, and 2.1 and 1.3 *ƞ*g/kg bw/day for elderly people. All the values obtained for P75 were below 1 ng/kg bw/day (0.001 *μ*g/kg bw/day) which is the health-based reference value established for AFs by international scientific expert committees: the Joint Expert Committee on Food Additives (JECFA) and Scientific Committee for Food (SCF) [36, 37]. This was not the case for the P95 values which were above the limit for teenagers and adults, suggesting that the risk is statistically higher for few of them. Mean, P75, and P95 values respecting this limit were obtained whatever the age group when considering eggs. The calculation of the AFB_1_ MOE, and their comparison to the related standard (100 for high exposure and 600 for save exposure, the closer the value to 600, the safer the level of exposure and vice versa) [38] clearly shows a higher exposure to AFB_1_ through chicken consumption. Mean MOE values were globally higher or around 600 with eggs, while with chicken it was also the case except for elderly people with an MOE value of 316 (risky). Indeed, AFB_1_ in food shall obey to the ALARA principle. Ananditya et al. [39] also reported the estimated daily intake (EDI) lower to the health-based reference value of 1 *ƞ*g/kg bw/day but MOEs showing an important risk in Indonesia. This may be explained by the fact that limits of MOE were defined based on animal studies which can often be misleading as the animals may be more resistant to aflatoxins than humans [40]. In the case of OTA, the estimated dietary daily exposures through the consumption of chicken and eggs varied between 0.5–2 *ƞ*g/kg bw/day and 0.5–1.6 *ƞ*g/kg bw/day, respectively (Table 4). This suggests a weekly intake lower than the provisional tolerable weekly intake of OTA for humans which is 100 and 120 *ƞ*g/kg bw/day as recommended by the Joint FAO/WHO Expert Committee on Food Additives (JECFA) and the European Food Safety Authority (EFSA), respectively [20, 33]. However, the associated MOEs were below the recommended 10,000 [20, 33], therefore suggesting that the risk shall not be eliminated. On the other side, food processing is known to impact mycotoxin contamination [41], and then this aspect should be taken into account while analysing the risk associated with ready-to-eat chicken.

## 4. Conclusion

Chicken and egg consumers in urban cities of Cameroon are not aware of mycotoxins and their potential health risk. The presence of AFs, AFB_1_, and OTA in these poultry products globally respects the limits, but a health risk should not be underestimated based on the populations' consumption frequency. A total diet study as well as the influence of local cooking processes' impact on mycotoxin content will be required before confirming this exposure.

## Figures and Tables

**Figure 1:** Map of Cameroon and its 10 regions with the pointed out 03 selected study areas.

**Table 1:** Descriptive statistics of data collected from the households' survey in the selected Cameroon urbanized areas (*N* = 900).

Variable		Total population	Centre	Littoral	West
*HH composition*					
HH respondents	Female (*n* (%))	552 (61.3)	210 (70.0)	186 (62.0)	156 (52.0)
	Male (*n* (%))	348 (38.7)	90 (30.0)	114 (38.0)	144 (48.0)
Total people, *n*		4705	1565	1582	1558
Children, 4–12 y (*n* (%))		1293 (27.5)	470 (30.0)	410 (25.9)	413 (25.5)
Teenagers, 13–19 y (*n* (%))		1766 (37.5)	520 (33.2)	610 (38.6)	636 (40.8)
Adult, 20–59 y (*n* (%))		1311 (27.9)	475 (30.4)	422 (26.7)	414 (26.7)
Elderly, ≥60 y (*n* (%))		335 (7.1)	100 (6.4)	140 (8.8)	95 (6.0)

*Education level of HH respondents (%)*					
No schooling		4.7	4.0	2.0	8.0
Primary		13.7	21.0	2.0	18.0
Secondary		34.3	34.0	54.0	15.0
University		47.3	41.0	42.0	59.0

*HH respondents' knowledge (%)*					
Fungal contamination		95.7	96.0	98.0	93.0
Mycotoxin contamination		23.0	6.0	11.0	52.0
Health risks associated with fungal contamination		18.0	23.0	2.0	29.0

*HH chicken consumption frequency (%)*					
Daily		41.0	45.0	36.0	42.0
Weekly^c^		13.7	15.0	12.0	14.0
Monthly^d^		30.0	25.0	34.0	31.0
Annually^e^		16.3	15.0	18.0	13.0

*HH egg consumption frequency (%)*					
Daily		69.0	65.0	70.0	72.0
Weekly^c^		17.0	18.0	17.0	16.0
Monthly^d^		9.3	12.0	8.0	8.0
Annually^e^		4.7	5.0	5.0	4.0

HH: households; ^c^just once/week; ^d^at least once/ month; ^e^at least once/year.

**Table 2:** Body weight and global amounts of chicken and eggs consumed as per age groups among the studied population of the selected Cameroon urbanized areas.

Household member	Corresponding age category (years old)	Body weight (kg)	Global amount consumed for the three regions (g/day)											
			Chicken						Eggs					
			Mean	Min	Max	P75	P90	P95	Mean	Min	Max	P75	P90	P95
Children	4–12	25.2 ± 5.2	12.5	0.07	60.1	10.5	58.4	60.1	15.5	0.09	69.2	21.8	56.1	69.2
Teenagers	13–20	56.3 ± 6.0	37.6	0.2	195.1	42.8	158.2	195.1	48	0.09	671.3	16.6	65.6	671.3
Adults	21–59	71.4 ± 10.2	27.3	0.1	158	31.6	109.5	158.0	17.8	0.09	97.4	23.1	67.1	97.4
Elderly people	≥60	76.9 ± 7.7	85.9	0.4	628.7	34.4	524.0	628.7	26.1	0.09	100.2	51.3	99.2	100.2

**Table 3:** Mycotoxin levels in samples of chicken feed, chicken tissues, and eggs collected at Cameroon urbanized areas.

Mycotoxins	Concentration (*η*g/kg)	Samples^*∗*^					
		LBBF	LBLF	IBLF	BBM	BBL	BLE
Total aflatoxins	Min	3900	3500	6900	1400	1800	700
	Mean ± SD	10300 ± 8242	6933.3 ± 4944	8233.3 ± 1258.3	1800 ± 200	1966.7 ± 208.2	966.7 ± 152.8
	Max	19700	12600	9400	2200	2500	1900
	P75	19700	12600	9400	2200	2500	1900
	P95	19700	12600	9400	2200	2500	1900

Aflatoxin B_1_	Min	3700	2700	3300	1000	700	800
	Mean ± SD	8200 ± 1200	5833.3 ± 4827.4	3600 ± 264.6	1233.3 ± 321.5	1033.3 ± 230.9	933.3 ± 57.7
	Max	19300	11400	3800	2000	1200	1100
	P75	19300	11400	3800	2000	1200	1100
	P95	19300	11400	3800	2000	1200	1100

Ochratoxin A	Min	800	800	1900	800	1000	1400
	Mean ± SD	1000 ± 173.2	933.3 ± 152.8	2233.3 ± 288.7	1400 ± 173.2	2266.7 ± 1000	1933.3 ± 208.2
	Max	1100	1000	2400	1700	4900	2000
	P75	1100	1000	2400	1700	4900	2000
	P95	1100	1000	2400	1700	4900	2000

^*∗*^LBBF: local bulk broiler feed; LBLF: local bulk layer feed; IBLF: imported bulk layer feed; BBM: broiler bulk muscle; BBL: broiler bulk liver; BLE: bulk layer egg.

**Table 4:** Total aflatoxins (AFT), aflatoxin B_1_ (AFB_1_), and ochratoxinA (OTA) daily intake related to chicken and egg consumption and associated exposure at Cameroon urbanized areas.

		Chicken					Eggs				
		AFT intake (*ƞ*g·kg^−1^·BW·day^−1^)	AFB_1_ intake (*ƞ*g·kg^−1^·BW·day^−1^)	MOE for AFB_1_	OTA intake (*ƞ*g·kg^−1^ BW·day^−1^)	MOE for OTA	AFT intake (*ƞ*g·kg^−1^.BW·day^−1^)	AFB_1_ intake (*ƞ*g·kg^−1^·BW·day^−1^)	MOE for AFB_1_	OTA intake (*ƞ*g·kg^−1^ BW·day^−1^)	MOE for OTA
Children	Min	0.005	0.003	127062.6	0.005	3506.9	0.003	0.003	120004.3	0.007	2586.7
	Mean	0.9	0.6	711.6	0.9	19.6	0.6	0.6	696.8	1.2	15.0
	Max	4.5	2.7	148.0	4.4	4.1	2.7	2.6	156.1	5.3	3.4
	P75	0.2	0.1	2964.8	0.2	81.8	0.05	0.04	9000.3	0.09	194.0
	P95	1.3	0.8	514.1	1.3	14.2	0.6	0.6	670.8	14.5	1.3

Teenagers	Min	0.007	0.004	99355.9	0.003	6093.8	0.002	0.001	268104.8	0.003	5778.9
	Mean	1.3	0.8	528.5	1.6	11.4	0.8	0.8	502.7	1.6	10.8
	Max	6.5	3.9	101.9	21.9	0.8	11.5	11.1	35.9	23.1	0.8
	P75	0.4	0.2	1684.0	0.1	261.2	0.04	0.03	11490.2	0.07	247.7
	P95	3.1	1.9	213.2	1.3	14.1	0.7	0.6	621.9	1.3	13.4

Adults	Min	0.003	0.002	252007.4	0.002	7728.2	0.001	0.001	340012.1	0.002	7328.9
	Mean	0.7	0.4	923.1	0.5	39.1	0.2	0.2	1719.2	0.5	37.1
	Max	4.2	2.5	159.5	2.5	7.1	1.3	1.3	314.2	2.6	6.8
	P75	0.2	0.1	2930.3	0.04	409.1	0.02	0.02	18000.6	0.05	388.0
	P95	3.2	1.9	207.1	1.2	15.0	0.6	0.6	660.9	1.3	14.2

Elderly people	Min	0.01	0.006	67854.9	0.01	1872.8	0.001	0.001	366203.6	0.002	7893.4
	Mean	2.1	1.3	316.0	2.0	8.7	0.3	0.3	1262.8	0.7	27.2
	Max	15.4	9.3	43.2	15.0	1.2	1.3	1.2	328.9	2.5	7.1
	P75	0.5	0,.3	1330.5	0.5	36.7	0.02	0.02	25352.6	0.03	546.5
	P95	1.5	0.9	430.1	1.5	11.9	0.02	0.02	21972.2	0.04	14.2

## Data Availability

Data used to support the findings of this study can be obtained upon request to the corresponding author.

## Abbreviations

ALARA: As low as reasonably achievable
EDE: Estimated daily exposure
EDI: Estimated daily intake
MOE: Margin of exposure
PTWI: Provisional tolerable weekly intake.
